The article "A rare case of tumefactive demyelination of brain: A case report and literature review" was retracted in 2026. Reasons: fabricated or falsified data; plagiarized data; plagiarized images; overlap with other authors' work.

# A rare case of tumefactive demyelination of brain: A case report and literature review

**DOI:** 10.1002/ccr3.8369

**Published:** 2023-12-21

**Authors:** Pugazhendi Inban, Ogbonnaya Akuma, Zenia Elavia, Chinaza Mercy Akuma, Mansi Singh, Meet Popatbhai Kachhadia, Agaba Barnett James Musiime

**Affiliations:** ^1^ Department of General Medicine Government Medical College Chennai India; ^2^ Ebonyi State University Abakaliki Nigeria; ^3^ Dr. DY Patil Medical College Pune India; ^4^ Nnamdi Azikiwe University Awka Nigeria; ^5^ Bogomolets National Medical University Kyiv Ukraine; ^6^ P.D.U Medical College, Civil Hospital Campus Rajkot India; ^7^ Royal College of General Practitioners (RCGP) London UK

**Keywords:** cerebral spinal fluid (CSF), magnetic resonance imaging (MRI), magnetic resonance spectroscopy (MRS), multiple sclerosis, tumefactive demyelination (TD), Wernicke's aphasia

## Abstract

This case report highlights the diagnostic challenges encountered in a 30‐year‐old female presenting with fever followed by Wernicke's aphasia without right‐sided weakness, ultimately diagnosed as tumefactive demyelination (TD). TD is a rare neurological condition often misidentified as brain tumors or inflammatory disorders. The case emphasizes the importance of precise differentiation through advanced magnetic resonance imaging, showing restricted diffusion at lesion edges and the absence of gadolinium enhancement. Accurate diagnosis is crucial for tailored treatment and prognostic assessment. This case contributes to our understanding of TD and underscores the need for continued research and collaboration in the field of rare neurological disorders.

## 1 INTRODUCTION

Multiple sclerosis is an infrequent inflammatory disease of the central nervous system (CNS) that is distinguished by its assorted clinical and radiological presentations.^1^, ^2^ Tumefactive demyelination (TD), or tumefactive multiple sclerosis, stands apart as a distinctive entity within this spectrum. Demyelinating lesions in the CNS are a sign of these diseases. These lesions can be big, measuring 2 cm or more in diameter, or small, measuring between 0.5 cm and 2 cm, but they have the potential to cause mass effects. This unique feature may result in these lesions being initially misidentified as tumor‐like space‐occupying lesions; however, they typically exhibit a characteristic appearance on radiographic imaging and are clinically benign.^3^, ^4^, ^5^ Tumefactive demyelination, which is distinct from multiple sclerosis, occurs at an estimated rate of about 1–2 per 1000 cases of MS, although some studies propose a higher incidence ranging from 1.4% to 8%.^6^, ^7^ However, tumefactive demyelinating lesions can occur concurrently with autoimmune diseases (e.g., Sjogren disease, lupus erythematosus, neuromyelitis optica), infectious diseases (e.g., Human Immunodeficiency Virus), malignancy (e.g., renal cell carcinoma), drug‐related conditions (e.g., tacrolimus, fingolimod), and postinfectious conditions (e.g., acute disseminated encephalomyelitis, acute hemorrhage leukoencephalitis). TD can show up on its own at the start of a disease or as other diseases progress, but the pathophysiology of how it happens is not well understood. On magnetic resonance imaging (MRI) scans, these lesions can appear either as a single large lesion or several lesions exhibiting varying degrees of contrast enhancement. We present here a case study involving a thirty‐year‐old female who presented with a fever lasting 3 days followed by Wernicke's aphasia without right‐sided weakness and whose MRI findings were consistent with tumefactive brain demyelination.

The article "A rare case of tumefactive demyelination of brain: A case report and literature review" was retracted in 2026. Reasons: fabricated or falsified data; plagiarized data; plagiarized images; overlap with other authors' work.

## 2 CASE PRESENTATION

We present a case of a 30‐year‐old female with a recent history of fever lasting for 3 days. She developed Wernicke's aphasia, which is characterized by difficulty understanding and producing spoken language without any associated weakness, 6 days after the fever started. The patient remained conscious throughout the course of her illness. No significant past medical history is noted.

Upon admission, a comprehensive physical examination was conducted. Vital signs, including blood pressure (120/80 mm Hg), heart rate (78 beats per minute), respiratory rate (16 breaths per minute), and oxygen saturation (98% on room air), fell within normal ranges, except for an elevated temperature of 38.5°C (101.3 F), likely due to a recent three‐day fever. The patient's general appearance was consistent with her stated age, and she exhibited no signs of acute distress. Notably, she remained alert and oriented throughout the examination, indicating her continued consciousness.

The neurological examination showed intact cranial nerve functions, normal muscle strength, and sensory function in all extremities, with no signs of ataxia or abnormal reflexes. However, the notable finding was the presence of Wernicke's aphasia, characterized by fluent but non‐meaningful speech, word‐finding difficulties, comprehension deficits, and impaired repetition. The rest of the neurological examination was normal. Examination of other systems revealed no significant abnormalities. The presence of Wernicke's aphasia suggested a potential neurological origin, warranting further diagnostic evaluation. Routine blood tests were normal. Inflammatory markers (erythrocyte sedimentation rate/C reactive protein (ESR/CRP)) and an autoimmune screen including autoantibodies, extractable nuclear antigen, double‐stranded DNA, anti‐neutrophil cytoplasmic antibody, as well as serum angiotensin‐converting enzyme (ACE), were also normal. Based on clinical exam findings and laboratory results that were within normal limits, there was low suspicion for various infectious and inflammatory differentials such as tuberculosis, sarcoidosis, vasculitis, and malignancies.

The article "A rare case of tumefactive demyelination of brain: A case report and literature review" was retracted in 2026. Reasons: fabricated or falsified data; plagiarized data; plagiarized images; overlap with other authors' work.

A magnetic resonance (MR) brain scan was performed to investigate the neurological symptoms. The MR scan revealed mild diffusion restriction at the edges of certain brain regions, suggesting an alteration in water movement within the affected areas. Additionally, gadolinium contrast administration showed no enhancement, indicating the absence of active inflammation or vascular changes in the brain. Gradient echo (GRE) and susceptibility‐weighted imaging (SWI) were not included in the imaging assessment, as shown in Figure 1.

**FIGURE 1:** Multi‐contrast Magnetic Resonance Imaging (MRI) Showing Mild Diffusion Restriction at the Edges of Brain Lesions Across Fluid Attenuated Inversion Recovery (FLAIR) and T2‐weighted (blue arrows).

The T2‐weighted MRI exhibited mild diffusion restriction at the periphery of brain lesions, suggesting limited water molecule movement and potential pathology, possibly indicative of demyelinating disorders or altered tissue integrity. Despite concerns raised about neurological conditions, the absence of gadolinium enhancement in imaging results diminished the likelihood of active inflammation or vascular changes, lessening the possibility of an acute neurological condition. Elevated protein and low glucose levels in the cerebral spinal fluid (CSF) analysis, as shown in Table 1, imply potential neurological issues, necessitating additional clinical assessment and testing to establish a precise diagnosis and treatment plan.

**TABLE 1:** Cerebral spinal fluid (CSF) lab values.

Parameter	Patient value	Normal range
CSF Protein	54 mg/dL	15–45 mg/dL
CSF Glucose	50 mg/dL	60–100 mg/dL
CSF Cells	60 mm^3^	N/A (No Range)
Differential Count	P60% L40%	N/A (No Range)

In the cerebrospinal fluid (CSF), six oligoclonal bands (OCBs) were observed, but there were no OCBs detected in the serum. Additionally, there were no indications of neuroinfection present in the CSF.

Magnetic resonance spectroscopy (MRS) revealed normal levels of metabolites in the affected brain regions. Specifically, there would be no significant abnormalities in the concentrations of metabolites such as N‐acetyl aspartate (NAA), creatine, choline, and lactate, as shown in Figure 2.

**FIGURE 2:** MRS reveals normal metabolite levels in affected brain regions, providing clarity on NAA, creatine, choline, and lactate concentrations.

The article "A rare case of tumefactive demyelination of brain: A case report and literature review" was retracted in 2026. Reasons: fabricated or falsified data; plagiarized data; plagiarized images; overlap with other authors' work.

Based on the clinical presentation and diagnostic findings, this case appears to be consistent with tumefactive demyelination; the absence of gadolinium enhancement indicates that there is no active inflammation or vascular changes. This normal MRS profile would further support the diagnosis of tumefactive demyelination, as it would not show the characteristic changes seen in other conditions like tumors or acute inflammation, aligning with the absence of gadolinium enhancement in the MRI findings.

The patient underwent a five‐day course of intravenous methylprednisolone at a daily dose of one gram and was subsequently switched to a tapering regimen of prednisone. Following this treatment, she was discharged in a stable neurological condition and admitted to inpatient rehabilitation, where the plan was to initiate immunomodulatory therapy on an outpatient basis. A review of the patient's medical records 4 months later indicated that she has been progressing favorably. At present, she is actively participating in speech therapy sessions aimed at enhancing her mild language‐related challenges, which include improvements in auditory comprehension, verbal expression, and thought organization.

We recommended that the patient be closely monitored and additional neurological assessments that may be necessary to determine the extent and progression of the demyelinating lesions be carried out. Additionally, ongoing support for the patient's language difficulties, such as speech therapy, may be beneficial in managing Wernicke's aphasia.

## 3 DISCUSSION

The presented case of a 30‐year‐old female with an initial presentation of fever for 3 days followed by the development of Wernicke's aphasia 6 days later, along with no right‐sided weakness, raises important diagnostic considerations. The patient is diagnosed with tumefactive demyelination (TD), and the aim of this case report is to shed light on the complex diagnostic challenges often encountered in the evaluation of this rare neurological condition. It emphasizes the crucial importance of precise differentiation in directing treatment approaches and, ultimately, enhancing patient outcomes. Our patient's case underscores the complexity involved in diagnosing TD.

Tumefactive demyelination typically presents with a wide range of acute neurological symptoms that may include focal deficits such as weakness, sensory disturbances, visual disturbances, and speech difficulties. Patients with TD may experience severe headaches, which can be mistaken for migraines or tension headaches. TD can lead to cognitive and behavioral changes, including confusion, memory problems, and personality changes.^8^ Clearly, our patient initially presented with a fever and developed Wernicke's aphasia 6 days later. These non‐specific symptoms added complexity to the diagnostic procedure. Common differential diagnoses typically include brain tumors (such as multifocal glioma, metastatic lesions, and CNS lymphoma), brain abscess, tuberculoma, and various inflammatory conditions like sarcoidosis and Sjögren's syndrome.^9^, ^10^

In contrast to acute disseminated encephalomyelitis (ADEM), tumefactive demyelinating lesions typically do not have a post‐infective origin. Also, people with multiple sclerosis (MS) can sometimes get large tumefactive demyelinating plaques that look like these lesions. This is called tumefactive multiple sclerosis. However, people who first show up with a single tumefactive demyelinating lesion rarely go on to get MS.^5^, ^9^

The diagnostic challenge in our case was to distinguish TD from brain tumors, abscesses, and other inflammatory conditions. Tumefactive Multiple Sclerosis (TMS) with a large tumefactive demyelinating lesion on imaging is a rare occurrence. Traditional MRI may not be very effective in distinguishing TDL from primary brain neoplasms or abscesses.^9^ Magnetic resonance (MR) may reveal specific characteristics that aid in the diagnostic process. Advanced magnetic resonance (MR) imaging of tumefactive demyelinating lesions reveals specific characteristics, including a high apparent diffusion coefficient, restricted diffusion at the periphery of the lesions, and low cerebral blood volume.^11^ Peripheral restriction is more common in inflammation and demyelinating disorders than in abscesses or tumors, whereas central restriction is specific to abscesses.^10^ Our patient had mild diffusion at the edges or periphery. This helped us to exclude tumors and abscesses. Nevertheless, despite these findings, diagnosis can be challenging, especially when a patient presents with a first neurological event and a solitary lesion on routine imaging.^9^ Notably, in suspected TMS cases, additional tests like CSF analysis for oligoclonal bands may not contribute significantly, as they are positive in only around 30% of TMS patients.^10^

The article "A rare case of tumefactive demyelination of brain: A case report and literature review" was retracted in 2026. Reasons: fabricated or falsified data; plagiarized data; plagiarized images; overlap with other authors' work.

The next diagnostic test that was done was gadolinium contrast. On imaging, TD shows absent or mild enhancement, indicating preserved blood–brain barriers. The absence of gadolinium enhancement also suggests that there is no active inflammation or vascular changes.^10^, ^12^ Our patient's diagnostics were negative for gadolinium contrast, ruling out any active inflammation.

In recent times, proton MR spectroscopy, employing cerebral biochemical substrate quantification, has emerged as a valuable non‐invasive diagnostic tool for delineating tumefactive brain lesions.^9^ MR spectroscopy has the capability to differentiate the presence and relative amounts of various chemical metabolites in the brain, making it a useful technique for further assessment of various intracranial diseases. It is particularly beneficial in determining the major category of disease manifested by the observed lesion, such as neoplastic, inflammatory, or ischemic. A neoplastic profile typically includes an attenuated NAA peak, indicative of neuronal loss; an elevated Cho resonance, suggesting increased turnover of cell membrane and myelin components; a reduced Cr peak, reflecting depressed cellular energetics and/or cell death from lesional necrosis; and, in some cases, detectable Lip and Lac peaks, signifying areas of cellular necrosis with the release of free lipids and anaerobic metabolism resulting in lactate production.^13^, ^14^ Elevation of lactate and choline peaks together, possibly explained by reactive astrogliosis, demyelination, and inflammation, leading to cell membrane breakdown, and reduction of NAA peak due to neuronal destruction, axonal damage, and neuronal mitochondrial dysfunction, are suggestive of demyelination.^14^ However, lactic peak is not specific to TMS.^14^ Despite the potential of MR spectroscopy, the existing literature, marked by study design heterogeneity, variable imaging timing, and a lack of histopathological data, remains insufficient to provide a definitive guideline for the use of MRS in clinical practice as a diagnostic tool.^9^ Further studies involving larger patient groups and standardized protocols are advisable before the full clinical utility of the technique can be determined.

In summary, this case underscores the complexity of diagnosing rare neurological conditions like TD. On MRI scans, the unique pattern of restricted diffusion at the edges makes TD different from brain tumors and abscesses. Negative gadolinium contrast makes TD different from any active inflammatory disorders, which shows how important it is to make a clear distinction. An accurate diagnosis is essential for customizing suitable treatment approaches, addressing patient expectations, and assessing the prognosis effectively.

In an era of advancing medical knowledge, dedication to research and clear communication among healthcare professionals continue to be crucial in enhancing outcomes for patients dealing with such conditions. This case adds to the expanding pool of information related to TD, underscoring the ongoing requirement for exploration and cooperation in the realm of rare neurological disorders.

The article "A rare case of tumefactive demyelination of brain: A case report and literature review" was retracted in 2026. Reasons: fabricated or falsified data; plagiarized data; plagiarized images; overlap with other authors' work.

## 4 CONCLUSION

Tumefactive demyelination, a rare neurological condition, often mimics brain tumors or inflammatory disorders, making accurate differentiation crucial for tailored treatment and improved outcomes. By presenting this case report, we aim to raise awareness about rare neurological manifestations, such as TD and we primarily focused on how we can rule out any other conditions such as brain tumors, abscesses, and active inflammatory conditions. It underscores the significance of including these rare and atypical presentations in the list of potential diagnoses. Moreover, we anticipate that our case report will address the paucity of literature regarding this demyelinating disorder, potentially catalyzing further research efforts to develop a more comprehensive diagnostic method and simplifying the differential diagnosis pathway.

## AUTHOR CONTRIBUTIONS

**Pugazhendi Inban:** Writing – original draft. **Ogbonnaya Akuma:** Writing – original draft. **Zenia Elavia:** Investigation. **Chinaza Mercy Akuma:** Resources. **Mansi Singh:** Writing – review and editing. **Meet Popatbhai Kachhadia:** Data curation. **Agaba Barnett James Musiime:** Methodology.

## FUNDING INFORMATION

None.

## CONSENT

Written informed consent was obtained from the patient to publish this report in accordance with the journal's patient consent policy.

## Data Availability

The datasets analyzed during the current study are available from the corresponding author upon reasonable request. Additionally, comprehensive literature sources used for the literature review are cited appropriately within the manuscript.
